# Protumor Effects of Histone H3–H4 Chaperone Antisilencing Feature 1B Gene on Lung Adenocarcinoma: In Silico and *In Vitro* Analyses

This article has been retracted.

**DOI:** 10.1155/2021/5005459

**Published:** 2021-12-16

**Authors:** Liyang Wu, Bing Jie

**Affiliations:** ^1^Affiliated Cancer Hospital & Institute of Guangzhou Medical University, Guangzhou Municipal and Guangdong Provincial Key Laboratory of Protein Modification and Degradation, State Key Laboratory of Respiratory Disease, School of Basic Medical Sciences, Guangzhou Medical University, Guangzhou, Guangdong 510095, China; ^2^Radiology Department, Shanghai Pulmonary Hospital, Affiliated with Tongji University, Shanghai, China

## Abstract

**Background:**

ASF1B is a member of the histone H3–H4 chaperone antisilencing feature 1 (ASF1). ASF1B reportedly acts as an oncogene in several cancers including, breast cancer and cervical cancer. To date, the role of ASF1B in lung adenocarcinoma (LUAD) is not elucidated.

**Methods:**

The TCGA database, containing data for 33 cancer types, was used to explore the dysregulation and prognostic value of the ASF1B gene in pan-cancer data. R software packages and public databases/webservers were applied for bioinformatics and statistical analyses. Using *in vitro* models, immunoprecipitation and immunofluorescence were utilized to investigate if BCAR1 interacted with ASF1B in LUAD. Further, transfection experiments were performed to validate the expression pattern of ASF1B in LUAD and examine its regulating role in tumor-associated processes including tumor cell proliferation and migration.

**Results:**

ASF1B was found to be significantly elevated in LUAD and the majority of cancer types, except PCPG (pheochromocytoma and paraganglioma). The overexpression of ASF1B was associated with worse prognostic outcomes in most cancer types including LUAD. ASF1B was associated with lymph node metastasis, and *in vitro*, it promoted the proliferation and migration of LUAD cells. ASF1B knockdown suppressed LUAD cell proliferation and migration and also diminished the expression of cell cycle, metastasis, and EMT signaling-associated proteins. BCAR1 was found positively correlated and interacting with ASF1B, and BCAR1 overexpression reversed the effects of ASF1B knockdown in LUAD cells.

**Conclusion:**

These findings indicated that ASF1B plays a significant role in the tumor progression of LUAD and BCAR1 mediates the tumor-promotive effects of ASF1B, acting as an intermediate protein. Therefore, the ASF1B/BCAR1 axis might be regarded as a putative therapeutic target for LUAD.

## 1. Introduction

Lung cancer, a highly prevalent malignant tumor, causes significant mortality and morbidity worldwide [1]. Non-small cell lung cancer (NSCLC), which includes lung squamous cell carcinoma (LUSC) and lung adenocarcinoma (LUAD) as the two main types, accounts for more than 85% of all lung cancer cases. Surgical resection, chemotherapy, and radiation therapy are all commonly applied treatments for early-stage LUAD, but they all have unwanted side effects [2, 3]. Of late, personalized precision medicine or P4 medicine, which adopts therapeutic strategies based on patients' specific molecular profiles, has gained much clinical interest owing to the promise of improved efficacy [4]. In particular, patients with LUAD typically have a poor prognosis, with a reported 5-year survival rate of only 15.9 percent [2]. Therefore, it is imperative to advance precision medicine approaches for LUAD by the identification of molecular targets for clinical translation.

Histone H3–H4 chaperone antisilencing feature 1 (ASF1) is a key histone chaperone protein involved in chromatin-based cellular DNA replication, DNA damage repair, and transcription control [5–8]. ASF1A and ASF1B are two paralogs of ASF1 [6, 7]. ASF1A is primarily involved in DNA repair and cell ageing, while ASF1B is primarily involved in cell proliferation [6, 7]. Several reports have noted a significant role of ASF1B in cancer. Corpet et al. reported that the elevated ASF1B mRNA level was linked to the clinical status and disease outcome in breast cancer and further proposed that ASF1B as a potential biomarker of breast cancer detection and prognosis [9]. Elsewhere, Liu et al. identified that ASF1B could promote the proliferation and migration of cervical cancer cells, suggesting its utility as a prognostic marker in cervical cancer [10]. In prostate cancer, ASF1B was found highly upregulated [11]. Moreover, inhibition of ASF1B induced G1 arrest and anticell apoptosis and prevented clonal formation [11]. A recent bioinformatic analysis utilizing publicly available TCGA and GEO databases noted that ASF1B is overexpressed in LUAD and elevated ASF1B expression is correlated with an advanced tumor stage, showing a significant prognostic value [12]. However, the detailed mechanisms in this context remain to be uncovered.

Breast cancer antiestrogen resistance 1 (BCAR1/p130Cas) is a scaffold protein, which is reportedly overexpressed, and serves to promote tumor proliferation and metastasis in multiple cancer types including lung cancer, breast cancer, and liver cancer [13–17]. In lung adenocarcinoma, BCAR1 has been shown to play a carcinogenetic role in the formation and immune evasion of invasive CTCs by triggering EMT via RAC1 signaling and modulating CD274 expression by translocating BRD4-S [18–21]. Little is known about the potential role of the interaction between BCAR1 and ASF1B in LUAD.

Therefore, the present study is aimed at exploring the mechanisms of ASF1B involvement in the pathogenesis of LUAD and also explored the putative role of ASF1B-BCAR1 interaction in this context by applying bioinformatic analysis and *in vitro* verification experiments.

## 2. Materials and Methods

### 2.1. Expression of ASF1B in Pan-Cancer Data

RNAseq data from The Cancer Genome Atlas (TCGA) database (URL: https://portal.gdc.cancer.gov/) and The Genotype-Tissue Expression (GTEx) cohort in TPM (transcript per million) format were downloaded from the University of California Santa Cruz (UCSC) Xena Browser (URL: https://xenabrowser.net) [22, 23] and uniformly processed using the TOIL process. The mRNA expression levels of ASF1B in multiple cancers were analyzed using and visualized by using the “ggplot2” package (version 3.3.3) in R (version 3.6.3). Transcript mapped data were normalized to the TPM format and then log_2_ transformed. A total of 15,776 samples were used for unpaired sample analysis and 10,534 samples were used for paired sample analysis. The Mann–Whitney *U* test (Mann–Whitney Wilcoxon test or the Wilcoxon rank-sum test) was used for comparing the ASF1B mRNA expression levels in healthy control and tumor groups. For paired sample analysis, if the data satisfied the Shapiro-Wilk normality test (*P* > 0.05), a paired sample *t*-test was used.

### 2.2. Expression of ASF1B in LUAD Samples in the TCGA Database

Level 3 HT-seq data of LUAD patients in the FPKM format were downloaded from the TCGA database (URL: https://portal.gdc.cancer.gov/) and GTEx cohort data from the UCSC Xena Browser (URL: https://xenabrowser.net) [22, 23]. Samples lacking clinical information were removed. Thereafter, 594 samples containing 535 LUAD tumor samples and 59 healthy control samples were included for the subsequent analysis regarding TCGA-LUAD dataset. RNAseq data with FPKM (fragments per kilobase per million) format were normalized into TPM (transcripts per million reads) format and then log_2_ transformed. The mRNA expression levels of ASF1B in LUAD were analyzed and visualized by using the “ggplot2” package (version 3.3.3) in R (version 3.6.3). Unpaired and paired sample analyses were both performed. For paired data satisfying the Shapiro-Wilk normality test (*P* > 0.05), a paired sample *t*-test was used. Unpaired data not satisfying the normality test (*P* < 0.05) were analyzed using the Mann–Whitney *U* test (Wilcoxon rank sum test). In addition, the dysregulation of the ASF1B gene reported in studies concerning LUAD was also examined by using the “Oncomine” web server (URL: https://www.oncomine.org/resource/login.html).

### 2.3. ROC Curve Analysis of the Diagnostic Value of ASF1B mRNA Expression in LUAD

ROC curve analysis of ASF1B gene expression data was conducted by using the “pROC” package (version 1.17.0.1) and visualized using the “ggplot2” package (version 3.3.3) in R (version 3.6.3). The clinical status (LUAD tumor vs. normal) was used as the outcome parameter. The *x*-axis abscissa represents the false-positive rate (FPR), and the *y*-axis represents the true-positive rate (TPR). ROC curves with an area under the ROC curve (AUC) > 0.9 indicates high diagnostic test accuracy, 0.7–0.9 indicates moderate accuracy, 0.5–0.7 indicates low accuracy, and 0.5 indicates a random result.

### 2.4. Tumor Clinical Characteristics of TCGA-LUAD Samples

Subsequent analysis was based on the TCGA-LUAD data obtained earlier. The expression levels of ASF1B mRNA, clinicopathological details, and general information pertaining to LUAD patients were obtained. Based on the median value of the ASF1B expression level, the LUAD samples were divided into two groups: a low-expression group of the ASF1B gene and a high-expression group of the ASF1B gene. The categorical variables analyzed included the TNM stage (T stage, N stage, and M stage), pathologic stage, primary therapy outcome, gender, race, age, residual tumor, anatomic neoplasm subdivision divided by the left or right sites, anatomic neoplasm subdivision divided by central/peripheral lung, smoking history including the number of pack years smoked, OS event, DSS event, and PFI event. If all levels of a certain categorical variable satisfied the conditions of theoretical frequency > 5 and total sample size > 40, the chi-square test was used; else, Fisher's exact test was applied for testing the differences between high- and low-LUAD expression groups. If the data for a certain categorical variable were not normally distributed (*P* < 0.05), the Wilcoxon rank sum test was used. Analysis was performed in R (version 3.6.3).

### 2.5. The Relationship between Tumor Clinical Characteristics and ASF1B Expression Levels

ASF1B mRNA expression levels in multiple clinical variable categories were analyzed. If the data of a certain clinical variable were normally distributed (*P* > 0.05), the Shapiro-Wilk normality test was used; otherwise, if the data of a certain clinical variable didn't satisfy the normality test (*P* < 0.05), the Kruskal-Wallis test was used. Such statistical analyses were performed and visualized by using the ggplot2 package in R program, based on the 329 LUAD tumor samples. In addition, the relationship between ASF1B expression and tumor characteristics was also investigated by applying a binary logistics model.

### 2.6. Survival Analysis

GEPIA (URL: http://gepia2.cancer-pku.cn/#index) was used to plot a survival map for ASF1B expression in pan-cancer data. The KM plotter web server (URL: https://kmplot.com/analysis/) was used to analyze the association between the ASF1B gene and the prognostic outcomes of LUAD tumor including overall survival (OS) and relapse-free survival (RFS).

### 2.7. Survival Analysis by Univariate and Multivariate Cox Regression

The association between tumor characteristics and prognosis was investigated by performing univariate and multivariate Cox regression analyses. The Cox-ph function in the “survival” package (version 3.2-10) in R (version 3.6.3) was applied and the cox regression module was used. The outcome selected was overall survival. The tumor characteristics included the T stage, N stage, M stage, pathologic stage, primary therapy outcome, gender, race, smoking status, age, number of pack years smoked, anatomic neoplasm subdivision, anatomic neoplasm subdivision, and ASF1B gene expression group.

### 2.8. Forest Plots

Based on the results (HR, 95% CI, *P* value) obtained from univariate and multivariate Cox regression analysis, two forest plots were plotted using the “ggplot2” package (version 3.3.3) in R (version 3.6.3). Each HR (hazard ratio) represents a relative risk of death that compares one level of a binary feature to the reference level. An HR > 1 indicates an increased risk of death, while an HR < 1 represents a decreased risk of death.

### 2.9. Identification of the Correlated Genes of ASF1B in LUAD

Gene correlation analysis for ASF1B was performed using the “stat” package (version 3.6.3) in R (version 3.6.3). The Pearson correlation test to assess the linear relationship between the two groups was applied, and only protein coding genes were retained. The cor-pearson value or the Pearson correlation coefficient “*r*” was obtained. A cor-pearson value of 0.90–1.00 indicates very strong correlation; 0.70–0.89 indicates strong correlation; 0.40–0.69 indicates moderate correlation; 0.10–0.39 indicates weak correlation; 0.00–0.10 indicates negligible correlation.

### 2.10. Heat map of ASF1B-BCAR Family Genes

The Cor-Pearson values of BCAR family genes (i.e., BCAR1, BCAR3, BCAR4, BCAR1P1, BCAR1P2, and BCAR3-AS1) were obtained. A heat map was plotted to show the expression pattern of these BCAR family genes in LUAD tumor samples. In addition, a scatter plot was visualized to depict the correlation between ASF1B and BCAR1. The “ggplot2” (version 3.3.3) package in R (version 3.6.3) was applied for this purpose.

### 2.11. Gene Set Enrichment Analysis

Genes with an absolute value of correlation coefficient > 0.1 and *P* value < 0.05 were used for gene set enrichment analysis (GSEA). Significant differentially expressed genes (DEGs) between LUAD and healthy control samples were identified by using “DESeq2” (version 1.26.0) in R (version 3.6.3) and based on the TCGA dataset. The log_2_FC (fold change) values for ASF1B significantly correlated genes were obtained and used for the gene set enrichment analysis (GSEA). GSEA analysis was performed using the “clusterProfiler” package (version 3.14.3) in R (version 3.6.3). Pathways were obtained from three databases including the KEGG pathway database, WikiPathways (WP) database, and Reactome (REAC). The referenced gene set was c2.cp.v7.2.symbols.gmt (Curated) in the MSigDB Collections (URL: https://www.gsea-msigdb.org/gsea/msigdb/collections.jsp#C2). Functional terms satisfying a condition of *P*.adjust < 0.05, false discovery rate (FDR) (also named *q* val) < 0.25, and ∣NES | >1 were considered as significantly enriched terms.

### 2.12. Functional Enrichment Analysis of Top 100 Significantly Correlated Genes of ASF1B

The top 100 genes ranked in a descending order of the cor_pearson value and the top 100 genes ranked in ascending order of the cor_pearson value were used for functional enrichment analysis to identify the significantly enriched functional terms among ASF1B-correlated genes. The gene names were converted to the Entrez ID by using the “http://org.Hs.eg.db” package (version 3.10.0) in R (version 3.6.3). Functional enrichment analysis was performed using the “clusterProfiler” package (version 3.14.3) in R (version 3.6.3). The species was selected as Homo sapiens and the Benjamini and Hochberg (BH) correction was applied to determine adjusted *P* values. GO terms including BP (biological process), CC (cellular component), and MF (molecular function) and KEGG pathways that were significantly enriched by the correlated genes were identified at a threshold of *P*.adj < 0.05 and *q* value < 0.2. If there were more than 30 terms, which were significantly enriched at this threshold setting, only the top 30 terms ranked in an ascending order of the adjusted *P* value were used to plot a bubble chart using “ggplot2” in R; otherwise, all of the terms were used.

### 2.13. Cell Lines and Culture

Non-neoplastic lung epithelial cell lines (HBE) and six LUAD cell lines (A549, H460, H1299, H1650, H1975, and PC9) were obtained from ATCC (American Type Culture Collection). Cells were cultured in RPMI-1640 medium (Thermo Fisher Scientific, USA) containing 10% fetal bovine serum (Gibco, USA) in an incubator at 37°C and 5% CO_2_.

### 2.14. siRNAs and Plasmid Transfection Experiments

siRNA targeting ASF1B and negative control were obtained from RiboBio (Guangzhou, China). Plasmids were purchased from Gene (Shanghai, China). siRNA and plasmid transfection was performed for ASF1B using Lipofectamine 3000 (Thermo Fisher Scientific Inc.) according to the manufacturer's instructions. In order to examine the effects of potential ASF1B-BCAR1 interaction in LUAD cells, firstly, ASF1B and BCAR1 were each overexpressed. Next, ASF1B knockdown was performed, followed by BCAR1 overexpression.

### 2.15. qRT-PCR

Total RNA was extracted using TRIzol RNA reagent (Thermo Fisher Scientific, USA). Reverse transcription was performed using the PrimeScript™ RT Reagent Kit with gDNA Eraser (TaKaRa, Japan). qRT-PCR was conducted using SYBR Green™ Premix Ex Taq™ II (TaKaRa, Japan) in an Applied Biosystems 7500 instrument (AB, USA). The primer sequence for each gene is described in Table S1.

### 2.16. Western Blot Analysis

Western blotting was performed according to a published protocol [24]. In brief, proteins were extracted in RIPA lysis buffer supplemented with phosphatase and protease inhibitors (CWBIO, Shanghai, China), and protein concentration was quantified with BCA Protein Assay (Thermo Scientific, Waltham, MA, USA). The proteins were separated by 10% SDS-PAGE and then transferred onto polyvinyl difluoride membranes (EMD Millipore, Billerica, MA, USA), followed by incubation with primary antibodies overnight. Primary antibodies used were as follows: *α*-tubulin, *β*-actin, ASF1B, BCAR1, Slug, CDK2/4, CCND1, P27 (CST), Snail, Slug, E-cadherin, and Vimentin (Abcam).

### 2.17. Immunoprecipitation (IP)

IP assay was performed to examine the possible binding between BCAR1 and ASF1B. IP was performed with the Pierce Co-Immunoprecipitation Kit (Thermo Scientific) according to the manufacturer's instructions. In brief, total proteins were extracted from cells and the amount of protein was quantified. After coupling the affinity-purified ASF1B antibody to amine- and carrier protein-free beads, proteins were incubated with the beads overnight at 4°C. The proteins were then pulled down with elution buffer, the samples were centrifuged, and the supernatant was collected. The samples were analyzed using mass spectrometry and Western blot. Anti-IgG (CST 2729S) was used as the negative control.

### 2.18. Immunofluorescence

Immunofluorescence was performed as previously described [24] to examine the colocalization of ASF1B with BCAR1. The cells were seeded on coverslips in 24-well culture plates and cultured overnight to facilitate attachment. After fixing in 4% paraformaldehyde, the cells were permeabilized in 0.2% Triton X-100 and then incubated with the indicated antibody overnight at 4°C. Cell nuclei were counterstained with 0.1 ml of DAPI (0.2 mg/ml), and the cells were visualized under a confocal microscope (Carl Zeiss, Germany). Antibodies included anti-ASF1B (Abcam, USA) and BCAR1 (ProteinTech, China).

### 2.19. Cell Counting Kit-8 (CCK-8) and Colony Formation Assays

Cells were plated into 96-well plates with 1000 cells per well. CCK-8 reagents (Djingo, Japan) were added at every at 24 h for five days. The optical density was estimated at 450 nm wavelength to assess cell viability. For colony formation assay, the cells were plated in 6-well plates (500/well) and incubated for 2 weeks at 37°C, 5% CO_2_. Colonies were washed thrice with PBS and stained with crystal violet for 15 min.

### 2.20. Wound Healing Assays

1 × 10^6^ cells were routinely seeded and inoculated in a 6-well plate. When the cell density reached 100%, scratching was performed with a 200 *μ*l sterile tip, perpendicularly to the cell plane. Photos were obtained under a microscope at the time points of 0 h and 24 h.

### 2.21. Migration Assays

Migration assays were performed using transwell chambers (Corning USA). For migration assays, cells (2 × 10^5^ cells) were seeded with serum-free medium onto the top chamber and the bottom chamber was filled with 10% FBS medium. After 18 h, cells in all the chambers were collected and fixed with methanol for 30 min, followed by staining with 0.01% crystal violet for 15 min.

### 2.22. Tumor-Immune Infiltrating Cells and Immune Genes Related to ASF1B Based on the Tumor Immune Estimation Resource Database

The “ESTIMATE” algorithm was applied, and calculated scores were downloaded from https://bioinformatics.mdanderson.org/estimate/. Precalculated TCGA data based on xCells was downloaded from xCells (http://xcell.ucsf.edu/).

### 2.23. Statistical Analysis

For data processing, GraphPad Prism version 8.0 was used. Values were presented as mean and SD (standard deviation) unless otherwise specified. For independent survey contrasts between two groups, when the two groups' SDs were equal, the Student's (two-tailed) *t*-test was used, and when the SDs were different, the Student's *t*-test with Welch's correlation was used. If the variances were equivalent in multigroup sample statistics, one-way ANOVA was used; if not, Welch's ANOVA was used. Both were subjected to Bonferroni post hoc testing. The TCGA LUAD cohort samples were split into two categories based on median gene expression values. Statistically significant differences were denoted as ^∗^*P* < 0.05, ^∗∗^ denotes *P* < 0.01, and ^∗∗∗^ denotes *P* < 0.0001.

## 3. Results

### 3.1. Dysregulation of ASF1B in Pan-Cancer Data and LUAD

To assess the role of ASF1B in cancer, firstly, a pan-cancer analysis of ASFIB expression in the TCGA cancer cohort data was performed. The results depicted in Figures 1(a) and 1(b) show that ASF1B was significantly upregulated in 32/33 cancer types, except PCPG. The results presented in Figures 1(c) and 1(d) depict that ASF1B was abundantly overexpressed in LUAD tumor samples as compared to healthy control samples.  Figure 1(e) indicates that the diagnostic value of ASF1B expression to discriminate LUAD from controls was very high (AUC = 0.947 > 0.7).  Table 1 summarizes the expression of ASF1B in four different LUAD studies, showing that the expression levels of ASF1B in LUAD tumor samples were significantly higher as compared to healthy control samples.

### 3.2. The Prognostic Value of ASF1B for Pan-Cancer and LUAD Outcomes

The prognostic value of ASF1B expression for pan-cancer data was assessed using the TCGA prognostic data (Figures 2(a) and 2(b)). First, the association between ASF1B expression and OS in pan-cancer data was analyzed, which demonstrated that elevated ASF1B mRNA expression was associated with poor prognosis in ACC, KIRC, KIRP, LAML, LGG, LIHC, LUAD, MESO, PAAD, and UVM, but good prognosis in CESC, LUSC, and STAD. In case of RFS, overexpressed ASF1B was found correlated with a short recurrence time in ACC, KIRP, LGG, LIHC, LUAD, PAAD, PRAD, THCA, and UVM, but correlated with longer recurrence time in COAD and STAD. The Kaplan-Meier plotter was utilized to validate the prognostic value of ASF1B in LUAD and consistent with the former results; ASF1B expression was significantly associated with OS and RFS (Figures 2(c) and 2(d)). Moreover, the univariate and multivariate cox regression analyses were performed to validate whether ASF1B could serve as an independent prognostic biomarker in lung adenocarcinoma. The respective results showed that ASF1B can be regarded as a potential predictor for the prognostic outcomes of LUAD (Table 2, Figures 2(i) and 2(j)).

### 3.3. Correlation of ASF1B Expression with the Clinicopathological Features of LUAD

To analyze the possible roles of ASF1B in LUAD pathogenesis, the relationship between the mRNA expression levels of ASF1B and the clinicopathological tumor parameters were examined.  Table 3 presents the tumor characteristics of the TCGA-LUAD patients in low- versus high-expression level groups of the ASF1B gene, and Table 4 shows the association between clinicopathological features of LUAD with ASF1B mRNA expression. As seen in Figures 2(e) and 2(h), ASF1B mRNA expression was significantly associated with four tumor characteristic variables including the N stage, pathologic stage, primary therapy outcome, and number of pack years smoked. However, there was no significant association between ASF1B mRNA expression levels with other variables including the T stage, M stage, gender, age, race, smoker, and anatomic neoplasm subdivision.

### 3.4. The Functional Terms Enriched by ASF1B-Correlated Genes

As ASF1B was earlier found to predict lymph node metastasis of LUAD, this finding was validated by conducting gene set enrichment analysis, based on the TCGA LUAD cohort. The GSEA results showed that several functional terms were significantly enriched by ASF1B-correlated genes including the formation of beta catenin TCF transactivating complex, G2_M_checkpoints, ESR-mediated signaling, signaling by Wnt, signaling by Notch, signaling by Rho_GTPASES, cell cycle, and MAPK signaling pathway (Figure 3(a)). Functional enrichment analysis showed that ASF1B top 100 correlated genes were significantly enriched in several biological processes including reticulum response to cadmium ion, response to zinc ion, cellular response to metal ion, cellular response to copper ion (Figure 3(b)); two KEGG pathways, i.e., mineral absorption and ribosome (Figure 3(c)); several cellular components, i.e., focal adhesion, ribosome, cell-substrate adherens junction, and large ribosomal subunit (Figure 3(d)); and several molecular functions, i.e., heat shock protein binding, chaperone binding, ligand-gated calcium channel activity, and bile acid transmembrane transporter activity (Figure 3(e)).

### 3.5. ASF1B Interacts with BCAR1 in LUAD Cells

Correlation analysis of ASF1B with multiple BCAR family genes in LUAD was performed and as depicted in Table 5 and Figure 4(a); the mRNA expression of ASF1B in LUAD was significantly correlated with 4/6 BCAR family genes, among which BCAR1 was positively correlated with ASF1B (Figure 4(b)). *In vitro*, IP assay demonstrated an interaction between BCAR1 and ASF1B in A549 cells (Figure 4(c)), showing extensive colocalization of ASF1B and BCAR1 in the cytoplasm of A549 cells (Figure 4(d)). To clarify the regulatory relationship between ASF1B and BCAR1, ASF1B plasmid was transiently transfected into A549 and PC-9 cells to overexpress ASF1B. As shown in Figure 4(e), BCAR1 protein expression was increased in both cell lines overexpressing ASF1B, whereas the ASF1B protein level was also increased upon upregulating BCAR1 (Figure 4(f)). These results demonstrated that ASF1B and BCAR1 can mutually promote each other's expression at the protein level in LUAD.

### 3.6. Decreased ASF1B Inhibits Proliferation of LUAD Cells

ASF1B expression levels in six different LUAD cell lines and human bronchial epithelial cell lines were examined using Western blotting. The results indicated that ASF1B was highly expressed in six LUAD cell lines at the protein level, among which A549 and PC-9 showed the highest expression levels (Figure. S1A). Therefore, A549 and PC-9 were used for further experiments. qPCR and Western blotting results demonstrated that ASF1B siRNA significantly decreased the expression of ASF1B (Figure. S1B-D). Colony formation and CCK8 assay verified that knockdown of ASF1B significantly blocked the proliferation of A549 and PC-9 cells (Figures 5(a)–5(c)). The Western blot results indicated that knockdown of ASF1B inhibited cyclin-dependent kinases (CDKs) CDK2/4 and cyclin proteins CCND1, while increasing the expression of the CDK inhibitor (CKI) P21 and P27 (Figure 5(d)).

### 3.7. ASF1B Promotes Cell Migration in LUAD

Transwell migration assays and wound healing assays demonstrated that knockdown of ASF1B inhibited the ability of tumor cell migration in LUAD (Figures 6(a)–6(d)). ASF1B knockdown decreased the protein expression levels of epithelial-mesenchymal transition- (EMT-) associated markers N-cadherin, Vimentin, Snail, and Slug and increased E-cadherin (Figure 6(e)).

### 3.8. Overexpression of BCAR1 in ASF1B-Blocked LUAD Cells Restores Cell Proliferation

The previous results suggested that ASF1B suppressed BCAR1 expression, but whether BCAR1 contributes to the proliferation and promoting function of ASF1B in LUAD remained unclear. Therefore, BCAR1 was overexpressed in A549 and PC-9 cells with ASF1B blocked, which led to enhanced LUAD cell proliferation as indicated by colony formation and CCK8 assays (Figures 7(a)–7(d)). In addition, the Western blot results indicated that CDK2/4 were restored, while P21 and P27 were attenuated (Figure 7(e)).

### 3.9. Overexpression of BCAR1 in ASF1B-Blocked LUAD Cells Promotes Cell Migration and Invasion

Further, it was investigated if BCAR1 was implicated in the metastasis-promoting effects of ASF1B on LUAD. When BCAR1 was restored in the two ASF1B knockdown LUAD cell lines, cell migration and invasiveness were restored as depicted by wound healing and transwell assays (Figures 8(a)–8(d)). Simultaneously, overexpressed BCAR1 markedly reversed the inhibition of EMT-related markers in ASF1B-obstructed LUAD cells (Figure 8(e)). These data proved that ASF1B mediated its metastasis promotive effects in LUAD by regulating BCAR1.

### 3.10. Correlation Analysis between ASF1B Expression and Immune Infiltration

The role of ASF1B in regulating the LUAD immune and tumor microenvironment is not known, so we tested the correlation between ASF1B expression and immune scores. ASF1B expression exhibited no significantly correlation with the stromal score, immune score, and ESTIMATE score in LUAD patients (Figure. S1E). We further examined the association between ASF1B and 64 noncancerous cell types to identify the crucial cellular components that participate in ASF1B-associated immunological processes. Our results demonstrated that 44 cell types were significantly associated with ASF1B, among which 22 cells were positively correlated, whereas 22 were negatively correlated (Table 6). Among these, CD8+ naive T cells and CD4+ naive T cells showed a strong correlation with ASF1B expression suggesting that ASF1B might be associated with tumor-infiltrating immune cells in LUAD and implicated in mediating immune escape mechanisms and regulation of the LUAD tumor microenvironment.

## 4. Discussion

Limitless replicative potential and tissue invasion and metastasis are two hallmarks of cancer [25], which are largely responsible for adverse prognosis. Considering the high clinical burden of LUAD, uncovering the molecular mechanisms of LUAD progression is of high priority to enable the discovery of highly effective therapeutic targets.

ASF1 is a member of the histone H3-H4 chaperone protein family that was first discovered in yeast [26]. ASF1A and ASF1B are the two members of ASF1, which controls chromatin functions and has been linked to tumorigenesis [5, 8, 9, 27], and its role has been investigated in prostate cancer, breast cancer, and cervical cancer [9–12]. Upregulated ASF1B expression has been associated with a higher risk of disease growth, cancer progression, and metastasis in small breast cancer [9]. Silencing ASF1B in prostate cancer blocked replication and cell cycle arrest and induced apoptosis, while knocking down ASF1B in cervical cancer was linked to proliferation, migration, and antiapoptosis effects [10]. Herein, bioinformatic analysis showed that ASF1B was overexpressed in most types of cancers including prostate and breast, supported by former research. In TCGA samples, overexpressed ASF1B was found associated with OS in 13/33 cancer types and RFS in 11/33 kinds of cancers, suggesting its putative value as a molecular biomarker of cancer prognosis. Here, we focused on deciphering the role of ASF1B in LUAD. Univariate and multivariate regression analyses depicted that the ASF1B mRNA expression level was an independent prognostic factor for OS in LUAD. In addition, ASF1B mRNA expression was significantly associated with lymph node metastasis and the clinical stage in LUAD. Applying gene set enrichment analysis, it appeared that ASF1B participated in G2_M_checkpoints, cell cycle, and signaling by Wnt, Notch, Rho-GTPases, and MAPK signaling pathways. These signaling pathways are classic pathways, which have been proved to regulate proliferation and metastasis in LUAD [28–31]. Besides, recent data has validated the findings of previous studies in breast cancer, prostate cancer, and cervical cancer [10]. As a result, it was conceived that ASF1B might play a role in LUAD proliferation and metastasis. *In vitro* experiments within the present study showed that the knockdown of ASF1B disrupted the proliferation of LUAD cells. Furthermore, blocking ASF1B with siRNA could inhibit migration of LUAD by reverse EMT *in vitro*, which was consistent with results noted in cervical cancer [10].

BCAR1 (also known as p130Cas/BCAR1) is an adaptor protein that belongs to the CAS family of scaffold proteins. Studies have clarified that BCAR1 is involved in carcinogenesis, by promotion of cell survival, growth, invasion, and migration. BCAR1 has been identified as a new promising biomarker for lung cancer [32]. Moreover, upregulated BCAR1 predicted poor prognosis in lung cancer patients and was associated with lymph node and distant metastasis and chemotherapy resistance in lung cancer [19, 20, 33, 34]. In order to explore the specific mechanism of the proliferation and metastatic promotion of ASF1B in LUAD, we first carried out a correlation analysis of ASF1B and BCAR family genes, showing that ASF1B was positively correlated with most of the BCAR family genes at the mRNA level and especially with BCAR1. Subsequently, we performed IP and immunofluorescence analyses, which depicted an interaction between ASF1B and BCAR1 in LUAD. In addition, the knockdown of ASF1B was accompanied by the decreased expression of BCAR1. Interestingly, BCAR1 has been widely reported to regulate the cell cycle and EMT in cancer [16, 20, 34]. Our current data indicated that ASF1B might promote cell proliferation and migration of LUAD by regulating cell cycle and EMT both. Hereafter, BCAR1 was overexpressed in LUAD cells with ASF1B blocked to further study the effect of ASF1B on BCAR1. The results showed that restored BCAR1 in ASF1B blocked LUAD cells restored the proliferation and migration attenuated by ASF1B silencing. Based on the above results, we concluded that ASF1B exerted its oncogene function by modulating BCAR1 in LUAD.

While the role of ASF1B has been reported in several cancers, the function of ASF1B in immune regulation in LUAD is poorly understood. Here, we focused on the putative relationship of the ASF1B expression level with immune scores and immune cell profiles in LUAD. ASF1B expression was found correlated with 44 types of noncancerous cells, including Th1/2 cells, which suggests its crucial role in regulating the tumor microenvironment. Overall, the present data contributes to the understanding of the function of ASF1B in tumor immunology and its use as a cancer biomarker in LUAD.

Our research is the first to uncover the role of ASF1B in the development and pathogenesis of LUAD. In sum, our findings indicate that ASF1B can be considered a relevant drug target and a prognostic biomarker in LUAD. Furthermore, these results also depict the plausible value of developing highly selective and active ASF1B inhibitors with a goal to counteract chemotherapy resistance and improve lung cancer treatment outcomes. However, preclinical and clinical studies that explore the comprehensive molecular mechanisms and signaling pathways involved in mediating the effects of ASF1B in LUAD are warranted.

## 5. Limitation

The present study did not include *in vivo* experiments to validate the role of ASF1B in the proliferation and metastasis of LUAD. In addition, gene enrichment analysis predicted that ASF1B as involved in the regulation of many classic pathways including MAPK, which has been shown to be regulated by BCAR1 [35]. Whether ASF1B regulates the proliferation and metastasis of LUAD through multiple signaling pathways remains to be investigated.

## Figures and Tables

**Figure 1:** The dysregulation of ASF1B in pan-cancer and LUAD data. The expression pattern of ASF1B in pan-cancer data analyzed using unpaired sample analysis (a) and paired sample analysis (b); the expression pattern of ASF1B in LUAD by using unpaired sample analysis (c) and paired sample analysis (d); ROC curve to evaluate the diagnostic value of ASF1B in discriminating LUAD from controls (e).

**Figure 2:** Prognostic value of ASF1B in TCGA pan-cancer and LUAD data. (a, b) Correlation between OS, RFS, and ASF1B mRNA expression in TCGA pan-cancer data. (c, d) Association between ASF1B gene expression and prognostic outcomes (overall survival (OS) and relapse-free survival (RFS)) of LUAD patients. The association between tumor characteristic variables ((e) N stage, (f) pathologic stage, (g) primary therapy outcome, and (h) Number_pack_years_smoked) and the expression level of ASF1B in LUAD. (h, i) Forest plot depicting results of univariate and multivariate analyses for OS as survival outcome.

**Figure 3:** The results of GSEA analysis and functional enrichment analysis. (a) The mountain plot showing the 28 functional terms with the top NES values; (b) the biological processes significantly enriched by the top 100 ASF1B-correlated genes; (c) the KEGG pathways significantly enriched by the top 100 ASF1B-correlated genes; (d) the cellular components significantly enriched by the top 100 ASF1B-correalted genes; (e) the molecular functions significantly enriched by the top 100 ASF1B-correlated genes.

**Figure 4:** ASF1B interacts and colocalizes with BCAR1 in LUAD. (a) Heat map showing the correlation between ASF1B and several BCAR family genes. (b) Scatter plot showing the correlation between ASF1B and BCAR1 in LUAD. (c) Binding between BCAR1 and ASF1B verified by immunoprecipitation. Cell lysates were immunoprecipitated with the anti-BCAR1 antibody. The input served as the positive control and IgG as the negative control. (d) Colocalization of ASF1B with BCAR1. Immunofluorescent signals for DAPI (blue) distributed in the nuclei. Green signals stand for ASF1B, and red signals represent BCAR1. The yellow signals indicate colocalization. (e) Western blot analysis of BCAR1 protein expression after ASF1B overexpression. (f) Western blot analysis of ASF1B protein expression after BCAR1 overexpression.

**Figure 5:** ASF1B promotes the proliferation of LUAD. (a, d) Colony formation assays, (b) CCK-8 assays depict that knockdown of ASF1B inhibits proliferation of LUAD cells. (c) Western blot analysis to evaluate the levels of proliferation signaling associated proteins' expression levels in LUAD.

**Figure 6:** ASF1B promotes migration of LUAD. (a, c) Wound Healing and (b, d) transwell assays demonstrated that ASF1B knockdown blocks the migration of LUAD cells. (e) Western blot analysis to examine metastasis signaling-associated protein expression levels in LUAD cells.

**Figure 7:** ASF1B promotes proliferation of LUAD via regulating BCAR1. (a, b) Colony formation assays. (c, d) CCK8 assays indicating induced BCAR1 in ASF1B knockdown A549 and PC9 cells restored cell proliferation ability. (e) Restoration of BCAR1 upregulated CDK2/4 and CCND1 and decreased P27 in ASF1B knockdown cells.

**Figure 8:** ASF1B promotes migration of LUAD cells by promoting BCAR1. (a, d) Wound healing. (b, c) Transwell assays depict increased migration ability after overexpressing BCAR1 in ASF1B knockdown LUAD cells. (e) Western blot results demonstrate decreased N-cadherin, Slug, Snail, Vimentin, and increased E-cadherin in ASF1B knockdown A549 and PC9 cells with BCAR1 overexpressed.

**Table 1:** Significant alterations of ASF1B expression at the transcriptional level in LUAD tissue and normal tissues (ONCOMINE database).

Source and/or reference	Fold change	*P* value	*t*-test
Garber Lung Statistics [37]	2.126	3.91*E* − 6	7.069
Su Lung Statistics [38]	2.305	3.28*E* − 8	6.678
Hou Lung Statistics [39]	2.257	1.89*E* − 14	9.633
Okayama Lung Statistics [40]	2.080	1.64*E* − 13	10.894

**Table 2:** Cox regression analysis for the association of overall survival of LUAD patients with clinical characteristics and the mRNA expression level of ASF1B.

Characteristics	Total (*N*)	Univariate analysis		Multivariate analysis	
		HR (95% CI)	*P* value	HR (95% CI)	*P* value
T stage (T3&T4 vs. T1&T2)	523	2.317 (1.591-3.375)	<0.001	2.256 (0.874-5.823)	0.093
N stage (N1&T2 vs. N0)	437	2.386 (1.698-3.352)	<0.001	1.716 (1.066-2.764)	0.026
M stage (M1 vs. M0)	377	2.136 (1.248-3.653)	0.006	1.856 (0.382-9.011)	0.443
Pathologic stage (stage III&stage IV vs. stage I&stage II)	518	2.664 (1.960-3.621)	<0.001	0.988 (0.271-3.604)	0.985
Primary therapy outcome (PD&SD vs. PR&CR)	439	2.653 (1.888-3.726)	<0.001	2.086 (1.281-3.395)	0.003
Gender (male vs. female)	526	1.070 (0.803-1.426)	0.642		
Race (Asian&Black or African-American vs. White)	468	0.678 (0.415-1.109)	0.121		
Smoker (yes vs. no)	512	0.894 (0.592-1.348)	0.591		
Age (>65 vs. ≤65)	516	1.223 (0.916-1.635)	0.172		
Number_pack_years_smoked (≥40 vs. <40)	363	1.073 (0.753-1.528)	0.697		
Anatomic neoplasm subdivision (right vs. left)	512	1.037 (0.770-1.397)	0.810		
Anatomic neoplasm subdivision (peripheral lung vs. central lung)	182	0.913 (0.570-1.463)	0.706		
ASF1B expression (high vs. low)	526	1.503 (1.125-2.007)	0.006	1.643 (1.036-2.606)	0.035

**Table 3:** Clinical characteristics of the TCGA-LUAD patients in low and high ASF1B gene. Expression level groups.

Characteristic	Low expression of ASF1B	High expression of ASF1B	*P*
*n*	267	268	
T stage, *n* (%)			0.018
T1	104 (19.5%)	71 (13.3%)	
T2	129 (24.2%)	160 (30.1%)	
T3	22 (4.1%)	27 (5.1%)	
T4	10 (1.9%)	9 (1.7%)	
N stage, *n* (%)			0.007
N0	187 (36%)	161 (31%)	
N1	36 (6.9%)	59 (11.4%)	
N2	31 (6%)	43 (8.3%)	
N3	0 (0%)	2 (0.4%)	
M stage, *n* (%)			0.104
M0	184 (47.7%)	177 (45.9%)	
M1	8 (2.1%)	17 (4.4%)	
Pathologic stage, *n* (%)			0.002
Stage I	167 (31.7%)	127 (24.1%)	
Stage II	50 (9.5%)	73 (13.9%)	
Stage III	35 (6.6%)	49 (9.3%)	
Stage IV	9 (1.7%)	17 (3.2%)	
Primary therapy outcome, *n* (%)			0.038
PD	25 (5.6%)	46 (10.3%)	
SD	20 (4.5%)	17 (3.8%)	
PR	3 (0.7%)	3 (0.7%)	
CR	178 (39.9%)	154 (34.5%)	
Gender, *n* (%)			0.241
Female	150 (28%)	136 (25.4%)	
Male	117 (21.9%)	132 (24.7%)	
Race, *n* (%)			0.936
Asian	3 (0.6%)	4 (0.9%)	
Black or African-American	28 (6%)	27 (5.8%)	
White	210 (44.9%)	196 (41.9%)	
Age, *n* (%)			0.028
≤65	115 (22.3%)	140 (27.1%)	
>65	144 (27.9%)	117 (22.7%)	
Residual tumor, *n* (%)			0.220
R0	168 (45.2%)	187 (50.3%)	
R1	6 (1.6%)	7 (1.9%)	
R2	0 (0%)	4 (1.1%)	
Anatomic neoplasm subdivision, *n* (%)			0.802
Left	104 (20%)	101 (19.4%)	
Right	155 (29.8%)	160 (30.8%)	
Anatomic neoplasm subdivision 2, *n* (%)			0.415
Central lung	31 (16.4%)	31 (16.4%)	
Peripheral lung	54 (28.6%)	73 (38.6%)	
number_pack_years_smoked, *n* (%)			0.106
<40	102 (27.6%)	86 (23.3%)	
≥40	82 (22.2%)	99 (26.8%)	
Smoker, *n* (%)			0.709
No	35 (6.7%)	40 (7.7%)	
Yes	222 (42.6%)	224 (43%)	
OS event, *n* (%)			0.006
Alive	187 (35%)	156 (29.2%)	
Dead	80 (15%)	112 (20.9%)	
DSS event, *n* (%)			0.002
Alive	204 (40.9%)	175 (35.1%)	
Dead	44 (8.8%)	76 (15.2%)	
PFI event, *n* (%)			0.031
Alive	167 (31.2%)	142 (26.5%)	
Dead	100 (18.7%)	126 (23.6%)	
Age, median (IQR)	67 (60, 74)	64 (57, 71)	0.002

**Table 4:** Logistic regression analysis outcomes showing the association of ASF1B expression with the clinical characteristics of LUAD patients.

Characteristics	Total (*N*)	Odds ratio (OR)	*P* value
T stage (T3&T4 vs. T1&T2)	532	1.135 (0.682-1.896)	0.627
N stage (N1&N2&N3 vs. N0)	519	1.803 (1.245-2.624)	0.002
M stage (M1 vs. M0)	386	2.209 (0.957-5.533)	0.073
Pathologic stage (stage III&stage IV vs. stage I&stage II)	527	1.628 (1.065-2.507)	0.025
Primary therapy outcome (PD&SD vs. PR&CR)	446	1.614 (1.044-2.512)	0.032
Gender (male vs. female)	535	1.244 (0.886-1.750)	0.208
Race (Asian&Black or African-American vs. White)	468	1.071 (0.626-1.832)	0.800
Age (>65 vs. ≤65)	516	0.667 (0.471-0.943)	0.022
Smoker (yes vs. no)	521	0.883 (0.539-1.441)	0.618
Residual tumor (R1&R2 vs. R0)	372	1.647 (0.613-4.871)	0.336
Anatomic neoplasm subdivision 2 (peripheral lung vs. central lung)	189	1.352 (0.734-2.493)	0.332
Number of pack years smoked (≥40 vs. <40)	369	1.432 (0.951-2.161)	0.086

**Table 5:** Correlation of ASF1B gene expression with BCAR family gene (e.g., BCAR1, BCAR3, BCAR4, BCAR1P1, BCAR1P2, and BCAR3-AS1) expression in LUAD.

gene_name	gene_id	gene_biotype	cor_pearson	p_pearson	cor_spearman	p_spearman
BCAR1	ENSG00000050820	protein_coding	0.162238804	0.000164025	0.140721599	0.001111262
BCAR3	ENSG00000137936	protein_coding	0.230477547	6.99727E-08	0.216999378	4.29962E-07
BCAR4	ENSG00000262117	lncRNA	0.135724142	0.001652162	0.092528582	0.032372662
BCAR1P1	ENSG00000258397	processed_pseudogene	0.061389195	0.156204593	0.068181393	0.115213758
BCAR1P2	ENSG00000258771	processed_pseudogene	0.00794493	0.854531382	0.01386953	0.74891663
BCAR3-AS1	ENSG00000224093	lncRNA	-0.164632803	0.00013067	-0.177556615	3.72916E-05

**Table 6:** Correlation of ASF1B with 64 types of noncancerous cell populations in LUAD.

xCells	Category	Pearson's *r* (95% CI)	*P* value
CD4+ memory T cells	Lymphoids	0.16 (0.07~0.24)	0.0005^∗∗∗^
CD4+ naive T cells	Lymphoids	−0.18 (−0.27~−0.10)	<0.0001^∗∗∗^
CD4+ T cells	Lymphoids	−0.06 (−0.14~0.02)	0.1553
CD4+ Tcm	Lymphoids	−0.23 (−0.31~−0.14)	<0.0001^∗∗∗^
CD4+ Tem	Lymphoids	−0.04 (−0.13~0.05)	0.3693
B cells	Lymphoids	−0.03 (−0.12~0.05)	0.4554
CD8+ naive T cells	Lymphoids	0.21 (0.13~0.30)	<0.0001^∗∗∗^
CD8+ Tcm	Lymphoids	0.08 (−0.00~0.17)	0.059
CD8+ Tem	Lymphoids	0.08 (−0.01~0.16)	0.0772
CD8+ T cells	Lymphoids	−0.03 (−0.12~0.05)	0.45
Class switched memory B cells	Lymphoids	−0.20 (−0.28~−0.11)	<0.0001^∗∗∗^
Memory B cells	Lymphoids	0.00 (−0.09~0.09)	0.9731
Naive B cells	Lymphoids	0.10 (0.013~0.19)	0.024^∗^
NK cells	Lymphoids	0.12 (0.03~0.21)	0.0064^∗∗^
Natural killer T cells (NKT)	Lymphoids	0.14 (0.06~0.23)	0.0012^∗∗^
Plasma cells	Lymphoids	0.03 (−0.06~0.12)	0.4852
Pro B cells	Lymphoids	0.31 (0.22~0.38)	<0.0001^∗∗∗^
Tgd cells	Lymphoids	0.05 (−0.03~0.14)	0.2193
Th1 cells	Lymphoids	0.62 (0.56~0.66)	<0.0001^∗∗∗^
Th2 cells	Lymphoids	0.53 (0.47~0.59)	<0.0001^∗∗∗^
Tregs	Lymphoids	0.03 (−0.06~0.11)	0.5347
Activated dendritic cells (aDC)	Myeloids	0.11 (0.02~0.19)	0.0176^∗^
Basophils	Myeloids	0.21 (0.13~0.30)	0.0002^∗∗^
Conventional dendritic cells (cDC)	Myeloids	−0.16 (−0.25~−0.08)	<0.0001^∗∗∗^
Dendritic cells (DC)	Myeloids	−0.09 (−0.18~−0.01)	0.0334^∗^
Eosinophils	Myeloids	−0.34 (−0.42~−0.26)	<0.0001^∗∗∗^
Immature DC (iDC)	Myeloids	−0.11 (−0.20~−0.02)	0.0124^∗^
Macrophages	Myeloids	0.10 (0.01~0.18)	0.0317^∗^
Macrophage M1	Myeloids	0.21 (0.12~0.29)	<0.0001^∗∗∗^
Macrophage M2	Myeloids	−0.23 (−0.31~−0.15)	<0.0001^∗∗∗^
Mast cells	Myeloids	−0.33 (−0.41~−0.25)	<0.0001^∗∗∗^
Monocytes	Myeloids	−0.00 (−0.09~0.08)	0.9245
Neutrophils	Myeloids	−0.02 (−0.11~0.06)	0.607
Plasmacytoid dendritic cells (pDC)	Myeloids	0.20 (0.12~0.29)	<0.0001^∗∗∗^
Astrocytes	Others	0.21 (0.12~0.29)	<0.0001^∗∗∗^
Epithelial cells	Others	−0.12 (−0.20~−0.03)	0.0077^∗^
Hepatocytes	Others	−0.10 (−0.19~−0.02)	0.021^∗^
Keratinocytes	Others	0.15 (0.06~0.23)	0.0008^∗∗^
Melanocytes	Others	0.02 (−0.07~0.11)	0.6831
Mesangial cells	Others	0.06 (−0.02~0.15)	0.1456
Myocytes	Others	−0.37(−0.44~−0.29)	<0.0001^∗∗∗^
Neurons	Others	0.08 (−0.00-0.17)	0.0596
Sebocytes	Others	−0.02 (−0.10~0.07)	0.6889
Common lymphoid progenitors (CLP)	Stem cells	0.32 (0.23~0.39)	<0.0001^∗∗∗^
Common myeloid progenitors (CMP)	Stem cells	−0.06 (−0.14~0.03)	0.217
Erythrocytes	Stem cells	0.14 (0.06~0.23)	0.0011^∗^
Granulocyte-macrophage progenitor (GMP)	Stem cells	−0.09 (−0.18~−0.00)	0.0432^∗^
Hematopoietic stem cells (HSC)	Stem cells	−0.61 (−0.67~−0.56)	<0.0001^∗∗∗^
Megakaryocytes	Stem cells	−0.40 (−0.47~−0.32)	<0.0001^∗∗∗^
Megakaryocyte-erythroid progenitors (MEP)	Stem cells	0.45 (0.38~0.52)	<0.0001^∗∗∗^
Multipotent progenitors (MPP)	Stem cells	−0.15 (−0.24~−0.07)	0.0005^∗∗^
Platelets	Stem cells	0.02 (−0.07~0.11)	0.6262
Adipocytes	Stromal cells	−0.29 (−0.37~−0.21)	<0.0001^∗∗∗^
Chondrocytes	Stromal cells	−0.33 (−0.40~−0.24)	0.0002^∗∗^
Endothelial cells	Stromal cells	−0.34 (−0.41~−0.26)	<0.0001^∗∗∗^
Fibroblasts	Stromal cells	−0.37 (−0.44~−0.29)	<0.0001^∗∗∗^
ly endothelial cells	Stromal cells	0.33 (0.25-0.40)	<0.0001^∗∗∗^
Mesenchymal stem cells (MSC)	Stromal cells	0.07 (−0.01~0.16)	0.0941
mv endothelial cells	Stromal cells	−0.19 (−0.27~−0.10)	<0.0001^∗∗∗^
Osteoblast	Stromal cells	0.17 (0.09~0.26)	<0.0001^∗∗∗^
Pericytes	Stromal cells	0.05 (−0.04~0.13)	0.2855
Preadipocytes	Stromal cells	−0.09 (−0.18~−0.01)	0.0378^∗^
Skeletal muscle	Stromal cells	0.12 (0.03~0.21)	0.0069^∗∗^
Smooth muscle	Stromal cells	0.24 (0.15~0.32)	<0.0001^∗∗∗^

LUAD: lung adenocarcinoma; ^∗^*P* < 0.05; ^∗∗^*P* < 0.01; ^∗∗∗^*P* < 0.001.

## Data Availability

The datasets used during the present study are available from the corresponding author upon reasonable request. Data were obtained from The Cancer Genome Atlas (TCGA; http://portal.gdc.cancer.gov) and the University of California Santa Cruz Xena Browser (https://xenabrowser.net).

## Supplementary Materials

Supplementary Materials Figure. S1: ASF1B expression in LUAD cells. (A) The protein expression ASF1B in six LUAD cell lines. (B-D) siRNA transfection blocked ASF1B expression at both mRNA and protein levels. (E) Correlation between ASF1B expression and the immune score, stromal score, and ESTIMATE score in LUAD patients. Table.S1: primers for RT-PCR.
